# Identification of a Ferroptosis-Related Prognostic Signature in Sepsis via Bioinformatics Analyses and Experiment Validation

**DOI:** 10.1155/2022/8178782

**Published:** 2022-05-25

**Authors:** Sizhe Zhu, Yabing Huang, Chenglin Ye

**Affiliations:** ^1^Department of Clinical Immunology, Tongji Hospital, Tongji Medical College, Huazhong University of Sciences and Technology, Wuhan, Hubei, China; ^2^Department of Pathology, Renmin Hospital of Wuhan University, Wuhan, Hubei, China

## Abstract

Ferroptosis is a new type of programmed cell death that is different from apoptosis, cell necrosis, and autophagy, which might be involved in development of sepsis. However, the potential role of ferroptosis-related genes (FRGs) in sepsis remained unclear. We identified 41 ferroptosis-related differential expression genes by weighted correlation network and differential expression analysis. The hub module of 41 ferroptosis-related differential expression genes in the protein-protein interaction network was identified. Next, we estimated diagnostic values of genes in hub modules. TLR4, WIPI1, and GABARAPL2 with high diagnostic value were selected for construction of risk prognostic model. The high risk-scored patients had significantly higher mortality than the patients with low risk scores in discovery dataset. Furthermore, the risk scores of nonsurvivor were higher than those of survivor in validation dataset. It suggested that risk score was significantly correlated to prognosis in sepsis. Then, we constructed a nomogram for improving the clinical applicability of risk signature. Moreover, the risk score was significantly associated with immune infiltration in sepsis. Our comprehensive analysis of FRGs in sepsis demonstrated the potential roles in diagnosis, prognosis, and immune infiltration. This work may benefit in understanding FRGs in sepsis and pave a new path for diagnosis and assessment of prognosis.

## 1. Introduction

Sepsis is defined as the host inflammatory response to life-threatening infections with organ dysfunction [1]. According to conservative estimates, sepsis is the leading cause of death and critical illness worldwide [2, 3]. Although the prognosis of sepsis has improved in the past few decades, the mortality rate with shock is still higher than 25%~30%, even 40%~50% [4]. Moreover, surviving sepsis patients usually have to suffer long-term physical, psychological, and cognitive impairments, and it has a significant impact on healthcare and society [5]. Furthermore, sepsis is differed from other major epidemics, the treatment of sepsis is nonspecific, and there are no approved drugs, but only through the support of organ function and the administration of intravenous fluids, antibiotics, and oxygen [6]. Therefore, there is an urgent need to explore new diagnostic and prognostic signature in sepsis.

Ferroptosis is an iron-dependent, nonapoptotic cell death method characterized by abnormal accumulation of lipid hydroperoxide and related lipophilic reactive oxygen species (ROS) in the cell membrane [7, 8]. Since the term was coined in 2012, the field of research on ferroptosis was grown exponentially in the past few years [9, 10]. Ferroptosis is involved in various pathological processes including neurotoxicity, acute kidney failure, liver injury, and heart disease, as well as myocardial ischemia reperfusion injury [11–14]. Furthermore, ferroptosis is related to sepsis and sepsis-induced organ injury. Inhibition of ferroptosis alleviates sepsis-induced acute lung injury [15]. Moreover, ferroptosis is involved in sepsis-induced cardiac injury [16]. Irisin suppresses ferroptosis in the liver of septic mice and restores mitochondrial function in experimental sepsis [17]. However, the comprehensive analyses in this filed are still needed.

In this work, we comprehensively evaluated the expression profiles of ferroptosis-related genes (FRGs) in sepsis. First, 936 sepsis patients from 6 independent Gene Expression Omnibus (GEO) datasets were included for further analyses. Three ferroptosis-related differential expression genes (FRDEGs) with high diagnostic value were selected for construction of risk prognostic model. Consequently, we established a scoring system to predict the likelihood of survival and characterize the immune infiltration of sepsis.

## 2. Methods

### 2.1. GEO Dataset Selection

The expression profile datasets of mRNAs were downloaded from the GEO (http://www.ncbi.nlm.nih.gov/geo) database. mRNAs from whole blood in human sepsis and healthy control were included. mRNA expression profiling data were obtained from GSE13904 (158 sepsis sample and 18 healthy control) [18] and GSE26378 (82 sepsis sample and 21 healthy sample) [19] datasets. Validation set were GSE80496 (21 sepsis sample and 21 healthy control) [20] and GSE134347 (156 sepsis sample and 83 healthy control) [21]. The prognostic value was investigated in GSE65682 as discovery dataset (468 sepsis sample with clinical information) [22], and GSE95233 (17 sepsis nonsurvivor and 34 survivor) was applied as validation dataset [23].

### 2.2. Differential Expression Analysis and Weighted Correlation Network Analysis

All analyses and visualization were performed in R version 3.6.3. Differential expression analysis was performed by limma R package [24], with adjusted *P* value < 0.05 and the log(fold − change) > 0.5 or <−0.5. Then, FRGs were downloaded from FerrDb, the world's first manually curated database for regulators and markers of ferroptosis and ferroptosis-disease associations (http://www.zhounan.org/ferrdb) [25]. Weighted correlation network analysis (WGCNA) is a widely used data mining method, and it is aimed at finding coexpressed gene modules (modules) and exploring the association between the gene network and the phenotype. WGCNA was applied to screen the relative modules in sepsis via WGCNA R package [26].The minimum number of module genes was set at 30. ParametersdeepSplit and mergeCutHeight were set at 3 and 0.25, respectively.

### 2.3. Gene Enrichment Analysis and Protein-Protein Interaction Network Construction

clusterProfiler R package was used for functional annotation of gene [27]. Gene Ontology (GO) and Kyoto Encyclopedia of Genes and Genomes (KEGG) pathway enrichment analyses were performed and visualized by ggplot2 R package [28]. The STRING database was used to construct the protein-protein interaction (PPI) network with medium confidence (0.4), and line color indicates the type of interaction evidence [29]. The hub genes were identified in EPC ranking method by Cytoscape and cytohubba [30].

### 2.4. Construction of 3 FRDEG Risk Models and Survival Analysis

To evaluate the diagnostic value of FRDEGs, receiver operating characteristic (ROC) curve was applied and area under the curve (AUC) was measured via pROC R package [31]. The least absolute shrinkage and selection operator (LASSO) regression was applied to construct a risk model via using the glmne R package [32]. The risk scores were calculated using the following formula: risk score = ∑_*i*=1_^*n*^coef∗*id* [33]. Survival analysis was performed by survminer and survival R packages. To estimate the likelihood of survival, a nomogram was constructed based on the risk score and clinical features by using the rms R package, and the prognostic ability of the nomogram was weighed by calibration plots.

### 2.5. Gene Set Enrichment and Immune Infiltration Analysis

Gene set enrichment analysis (GSEA) was performed via GSEA/MSigDB [34] and visualized by ggplot2 R package. CIBERSORT was applied to estimate the differential of immune cell infiltration in two groups [35].

### 2.6. Cecal Ligation Puncture Mouse Model

Beijing Vital River Laboratory Animal Technology Co. Ltd. provided 20 specific pathogen-free female C57BL/6J mice (8-10 weeks old, weighing 20-22 g). All animal experiments at Tongji Hospital were carried out in strict conformity with the Institutional Animal Care and Use Committees and the Institutional Review Board. The Medical Ethics Committee at Tongji Hospital expressly approved all mouse experimental procedures for this work, and they were carried out in compliance with institutional norms (TJ-IRB20182677) and the guidance for the care and use of laboratory animals (National Academies Press, 2011). All animal experiments met the ARRIVE guidelines [36]. All procedures on mice were performed under sodium pentobarbital anesthesia, and all efforts were made to minimize suffering. Cecal ligation puncture (CLP) mouse model is the most frequently used sepsis model, and protocol of CLP mouse model was referred to previous report with high-grade sepsis [37]. 12 h after surgery, the blood was collected from orbital sinus.

### 2.7. qRT-PCR

TRIpure Reagent was used to extract total RNA from blood of CLP mice, and the PCR conditions were 95°C for 5 min, followed by 40 cycles of 95°C for 15 s, 60°C for 15 s, and 72°C for 30 s. The relative gene expression level was calculated using the 2-*ΔΔ*Ct method. To normalize the data, GAPDH was used as internal reference. The sequences of the primer are shown in Table 1.

## 3. Results

### 3.1. Identification of FRDEGs

A flowchart of the study design is shown in Figure 1. Two sepsis public datasets, GSE13904 (*n* = 176) and GSE26378 (*n* = 103) were obtained from the GEO database. The limma R package was used for FRG differential gene expression analysis with thresholds of |Log2 (FC)| > 0.5 and adjusted *P* value < 0.05. A total of 56 and 70 FRDEGs were identified in GSE13904 and GSE26378, and results were presented in volcano plots, respectively (Figures 2(a) and 2(b)). WGCNA was applied to screen the relative modules, a threshold power of *β* = 14 was systematically selected to construct the scale-free network, while *R*^2^ cut at 0.86 (Figure 2(c)). As shown in Figures 2(d) and 2(e), WGCNA identified 16 modules, and steelblue and bisque modules have a strong positive (module trait correlation = 0.87) and negative (-0.80) connection to sepsis, respectively. The intersection of two groups of FRDEGs and steelblue as well as bisque modules is presented in Figure 2(f). Totally, 41 overlapped FRDEGs in red cycles were identified to further analyses.

### 3.2. Gene Enrichment Analysis and Protein-Protein Interaction Network Construction

GO and KEGG enrichment analyses were conducted, and top 10 biological process (BP) and KEGG pathways are shown in Figures 3(a) and 3(b). Terms of BP indicated that FRDEGs of sepsis were associated with response to starvation (*P* = 5.66*e* − 15), response to nutrient levels (*P* = 6.90*e* − 14), cellular response to external stimulus (*P* = 2.07*e* − 13), cellular response to extracellular stimulus (*P* = 3.27*e* − 13), and cellular response to starvation (*P* = 7.01*e* − 13). Top 3 of KEGG signaling pathways were autophagy–animal (*P* = 5.71*e* − 09), ferroptosis (*P* = 2.04*e* − 08), and FoxO signaling pathway (*P* = 7.99*e* − 08). The PPI network of 41 FRDEGs was constructed by the STRING database and visualized by Cytoscape which are shown in Figure 3(c). The hub module was identified by Cytoscape MCODE which is presented in Figure 3(d).

### 3.3. Validation of the Hub Genes in Sepsis

To validate the genes in hub clustering module, GSE80496 (*n* = 42) and GSE134347 (*n* = 239) were downloaded as validation set. ROC analyses of the genes were performed by pROC R package, and AUC was calculated to estimate the predictive performance. As shown in Figures 4(a) and 4(b) and Figure S1, TLR4, WIPI1, and GABARAPL2 had outstanding AUC (>0.90) in both two validation sets, reached 0.964, 0.988, and 0.975 in GSE80496 and 0.933, 0.961, and 0.964 in GSE134347, respectively. Moreover, the expressions of TLR4, WIPI1, and GABARAPL2 in two validation sets are exhibited in Figures 4(c)–4(h).

### 3.4. Construction of 3 FRDEG Risk Models and Survival Analysis

TLR4, WIPI1, and GABARAPL2 were used to create a risk model using LASSO regression (Figures 5(a) and 5(b)). The risk model was established to evaluate the survival risk for each patient as follows: risk score = 0.13749 × WIPI1 − 0.23614 × TLR4 + 0.40224 × GABARAPL2. We calculated each patients' risk score in GSE65682 datasets based on 3-gene signature. The median risk score was used to divide patients into high- and low-risk groups. Patients with a high risk score had a significantly higher mortality rate than those with a low risk score, as illustrated in Figure 5(c) (*P* = 4.3*e* − 3). To validate the 3-gene risk signature, the risk scores of sepsis nonsurvivor and survivor were estimated in validation dataset. As shown in Figures 5(d) and 5(e), sepsis nonsurvivors had significantly higher risk scores than survivors (*P* < 0.001), and AUC of risk score was 0.803. A nomogram was created to estimate the chances of survival in sepsis (Figure 6(a)). Nomogram forecasts with great accuracy, as illustrated in the calibration charts (Figures 6(b)–6(d)).

### 3.5. GSEA and Immune Infiltration Analyses

The differential of BP between high-risk and low-risk groups was explored by GSEA. As shown in Figure 7(a), the high-risk group significantly enriched in 3 gene sets with *P* value < 0.05, mainly reactome_neutrophil_degranulation, reactome_antimicrobial_peptides and reactome_innate_immune_system. In addition, the low-risk group enriched in reactome_interferon_signaling, reactome_interferon_alpha_beta_signaling, reactome_cytokine_signaling_in_immune_system (Figure 7(b)).

In consideration of the enrichment related to immune-related signaling pathways, the immune infiltration analysis was performed via CIBERSORT. The violin plot of the immune cell infiltration is presented in Figure 7(c). It is shown that the infiltrating levels of plasma cells, T cell CD4 naïve, T cell CD4 memory activated, T cell regulatory, NK cells resting, macrophage M0, macrophage M2, mast cells resting, and eosinophils were relatively upregulated in the high-risk group. Inversely, the fractions of B cell memory, mast cells activated, and neutrophils were relatively low in the high-risk group.

### 3.6. Validation of the Expression in CLP Mouse Model

CLP mouse model was used to simulate sepsis. As shown in Figures 8(a)–8(c), the relative expression of TLR4, GABARAPL2, and WIPI1 was measured via qRT-PCR. Importantly, the expression of TLR4, WIPI1, and GABARAPL2 was significantly upregulated in CLP mice. These results were consistent with the previous bioinformatics analyses.

## 4. Discussion

Sepsis remains one of the major causes of morbidity and mortality in critically ill patients [38]. Recent studies have shown that ferroptosis is involved in regulations of the occurrence and development of sepsis [16, 39]. However, the comprehensive analyses of the combined effects of multiferroptosis genes in sepsis are still needed.

In this work, comprehensive bioinformatics analyses were performed based on expression profile of sepsis from the GEO database. Furthermore, expression levels of FRGs were analyzed in sepsis datasets. A total of 41 FRDEGs were screened via differential analysis and WGCNA. Then, the hub module was identified in the PPI network, and the diagnostic values of FRDEGs in hub module were explored and verified. Therefore, 3 FRDEGs (TLR4, WIPI1, and GABARAPL2), with high sensitivity and specificity in sepsis diagnosis, were selected for construction of prognostic risk signature. Our results demonstrated that the risk scores of signature were significantly associated with prognosis. The high risk-scored patients had significantly higher mortality than the patients with low risk score. Consequently, a quantitative nomogram was established based on risk scores and ages, which can further improve the performance and facilitate the use of risk signature. Finally, the expression of genes in risk signature was also validated in CLP mouse model via qRT-PCR.

Sepsis is a complex interaction that triggers the host's proinflammatory and anti-inflammatory processes, and the balance of inflammatory and anti-inflammatory responses is vital. There are several studies showed that sepsis induces numerous overlapping mechanisms of immunosuppression involving both innate and adaptive immunity [40, 41]. The race to death in these immune mechanisms determines the fate of the septic patients. Therefore, in order to explore the underlying immune mechanisms, GSEA and immune infiltration analyses were performed. According to results of GSEA, the high-risk group was significantly enriched in pathway of neutrophil degranulation and innate immunes. It was reported that neutrophil degranulation resulted in iron-dependent accumulation of lipid peroxides, which promoted ferroptosis in glioblastoma [42]. Moreover, excessive neutrophil activation results in degranulation and release of reactive oxygen species into the extracellular medium, which leads to host tissue injury [43, 44]. Conversely, the interferon-related signaling pathway was enriched in the low-risk group, especially IFN-*α* and IFN-*β* pathway. IFN-*α* and IFN-*β* protected mice from LPS-induced lethality and septic shock in sepsis mouse model. These may explain the higher 4-week mortality in the high-risk group. The immune infiltration analysis showed that there was a differential between high- and low-risk groups. The fractions of neutrophil were relatively low in the high-risk group. Neutrophils are the most abundant cells in innate immunity, which are important for early controlling of invade pathogens. However, dysregulation of neutrophil migratory and activation correlates with the degree of clinical deterioration in patients with sepsis [45]. The number of NK cells is significantly decreased in septic patients, and it lasts for several weeks as well as it is associated with increased mortality [46–48]. Furthermore, the high-risk group had high infiltration level of T cell regulatory. It was consistent with the findings of previous studies, and increased percentage and number of T cell regulatory in peripheral blood are strongly associated with poor prognosis in patients with severe sepsis [49, 50]. The above results suggest that 3 FRDEGs might play an important role in prognosis and development of sepsis.

There are some limits. All sepsis cases were found from public databases in this retrospective analysis. As a result, we need larger datasets and prospective studies to back up our findings. Moreover, we failed to find another expression profiles of sepsis patient with 4-week survival data to further validation.

## 5. Conclusions

In summary, our comprehensive analyses revealed the potential roles of FRGs in sepsis. Furthermore, 3 FRDEGs had excellent diagnostic values. Importantly, FRDEG-based risk signature and nomogram could reliably predict prognosis of sepsis patients. Our work might highlight the crucial clinical implications of FRGs and provide novel insight into ferroptosis in sepsis.

## Figures and Tables

**Figure 1:** Flowchart of overall study design.

**Figure 2:** Identification of FRDEGs. (a, b) Volcano plots of differential genes in GSE13904 and GSE26378 with *P* value < 0.05, |log(fold − change)| > 0.5. (c) Determination of soft-thresholding power in WGCNA. (d) Clustering dendrogram in WGCNA. (e) The module-trait relationships in WGCNA. (f) A Venn diagram indicating overlapped FRDEGs between bisque module, steelblue module, GSE13904, and GSE26378 (circled in red).

**Figure 3:** Functional annotation of FRDEGs. (a) Top 10 GO enrichment; (b) top 10 KEGG enrichment; (c) the PPI network constructed via Cytoscape; green represents downregulated, and red represents upregulated genes; (d) hub clustering module identified by cytohubba.

**Figure 4:** Validation of TLR4, WIPI1, and GABARAPL2. (a, b) ROC curves and AUC of top 3 hub genes in GSE80496 and GSE13437; (c–h) the expression of TLR4, WIPI1, and GABARAPL2 in GSE80496 and GSE13437 (^∗∗∗^*P* < 0.001).

**Figure 5:** Construction and validation of risk signature. (a) In the LASSO model, ten-fold cross-validation for hub gene coefficients. (b) In the LASSO model, selection of optimal parameter (lambda). (c) A comparison of high- and low-risk groups' survival rates. (d) Risk ratings in validation datasets for sepsis survivors and nonsurvivors. (e) Risk score ROC curve (^∗∗∗^*P* < 0.001).

**Figure 6:** Construction and validation of a nomogram. (a) A nomogram to predict 1-, 2-, and 4-week survival. (b–d) The 1-, 2-, and 4-week nomogram calibration curves, respectively.

**Figure 7:** GSEA and immune infiltration analysis. (a) GSEA in the high-risk group; (b) GSEA in the low-risk group; (c) immune infiltration in high- and low-risk groups (^∗^*P* < 0.05, ^∗∗^*P* < 0.01, and ^∗∗∗^*P* < 0.001; ns: not significant).

**Figure 8:** The relative expression measured in CLP mice via qRT-PCR. (a) TLR4; (b) WIPI1; (c) GABARAPL2 (^∗∗∗^*P* < 0.001).

**Table 1:** The sequences of qRT-PCR primer.

Gene names	Primer sequence (5′-3′)
WIPI1	Forward-AGGATACTCTGAGGACGGCG Reverse-TCTGACTTCCACGGCACAAG

GABARAPL2	Forward-CCGTTGTTGTTGTGGTCGCT Reverse-TGAGAGCCCGAGACTTTTTCC

TLR4	Forward-TTTATTCAGAGCCGTTGGTG Reverse-CAGAGGATTGTCCTCCCATT

GAPDH	Forward-GCAAGTTCAACGGCACAG Reverse-GCCAGTAGACTCCACGACAT

## Data Availability

The datasets used to support the findings of this study are available from GEO (http://www.ncbi.nlm.nih.gov/geo) database. All data can be acquired from the corresponding authors on request.

## Supplementary Materials

Supplementary Materials Figure S1: validation of all hub genes. (A, B) ROC curves and AUC in GSE80496 and GSE13437.
